The article "The prognostic value of MGMT promoter status by pyrosequencing assay for glioblastoma patients’ survival: a meta-analysis" was published in 2016. Journal: World J Surg Oncol.

# The prognostic value of MGMT promoter status by pyrosequencing assay for glioblastoma patients’ survival: a meta-analysis

**DOI:** 10.1186/s12957-016-1012-4

**Published:** 2016-10-12

**Authors:** Hailong Zhao, Shuying Wang, Chengwei Song, Yunhong Zha, Li Li

**Affiliations:** 1 Department of Neurology, The First Hospital of Yichang, Institute of Translational Neuroscience, Three Gorges University College of Medicine, Yichang, People’s Republic of China; 2 Wuhan Institute of Biological Products Co., Ltd., Wuhan, People’s Republic of China

**Keywords:** MGMT, Meta-analysis, Glioblastoma, Hazard ratio, Pyrosequencing, Survival, Prognostic biomarker

## Abstract

**Background:**

The prognostic value of the status of O^6^-methylguanine-DNA methyltransferase (MGMT) promoter methylation measured by pyrosequencing assay (PSQ) among glioblastoma (GBM) patients was examined in meta-analysis.

**Methods:**

Eligible studies that reported the association between the status of MGMT promoter methylation by PSQ and prognostic value of GBM patients from three electronic databases, like PubMed, EMBASE, and Cochrane library were involved in meta-analysis. Using Stata 11.0, the summarized hazard ratios (HRs) for overall survival (OS) and the progression-free survival (PFS) with 95 % confidence interval (CI) were calculated.

**Results:**

Eleven studies were included to evaluate the relationship between the status of MGMT promoter methylation and GBM patients’ survival. Overall, regardless of the cut-off value of methylation status of MGMT promoter by PSQ, methylated-positive patients were evidently associated with an improved HRs for OS (HRs = 0.50, 95 % CI = 0.35–0.66). For summary, progression-free survival (PFS) from four studies, the prognostic effect was also found (HRs = 0.56, 95 % CI = 0.32–0.80).

**Conclusion:**

Methylation positivity of MGMT promoter by PSQ was related to an increased survival in GBM patients. Thus, the status of MGMT promoter methylation by PSQ might be used to be a prognostic biomarker, and GBM patients might have a vested interest in clinical application of standardized PSQ.

## Background

Glioblastoma (GBM), accounting for approximately 16 % of primary brain and central nervous system tumors in adults [1], has a poor prognosis with the median survival no more than 12 months [2], despite advances in chemotherapy, radiotherapy, surgery, and multi-modal treatments. A number of studies document that some molecular markers, such as IDH1/IDH2 [3], 1p/19q co-deletion [4], and MGMT promoter methylation [5], have become an integral part of tumor assessment in modern oncology practice. In 2016, the new World Health Organization (WHO) Classification of Tumors of the Central Nervous System (2016 CNS WHO) was launched to replace the 2007 CNS WHO. The new classification system integrates phenotypic and genotypic diagnoses, for example, GBM, on the basis of histological diagnosis, which is grouped into GBM IDH-wildtype, GBM IDH-mutant, and GBM NOS (not otherwise specified) with IDH mutational status; thus, patients will benefit from greater diagnostic accuracy as well as improved patient management and more accurate determinations of prognosis and treatment response [6]. Although classification has been established on the basis of IDH status among GBM, some studies indicated that IDH mutation, MGMT promoter methylation status, 1p/19q loss independently associated with favorable outcome in temozolomide (TMZ) + radiotherapy-treated GBM patients. Meanwhile, it was found that MGMT promoter methylation is a predictive marker for benefit from alkylating agents only in high-grade glioma patients with IDH1 wildtype, but 1p/19q loss in high-grade glioma patients with IDH1 mutant [7]. Nevertheless, in this meta-analysis, the predictive or prognostic role of MGMT promoter methylation among GBM was assessed.

The article "The prognostic value of MGMT promoter status by pyrosequencing assay for glioblastoma patients’ survival: a meta-analysis" was published in 2016. Journal: World J Surg Oncol.

MGMT, a DNA repair protein, removes the alkylation of the O^6^ position of guanine which is the most cytotoxic lesion induced by alkylating agent chemotherapy, such as nitrosoureas or temozolomide (TMZ) [8, 9]. Low-level expression of MGMT protein causes impaired ability to repair DNA. Hyper-methylation of MGMT gene promoter might result in silencing gene expression and further down-regulate protein concentrations [10]. Since a landmark study by Hegi [11] 11 years ago, numerous studies have confirmed that methylation status of MGMT promoter can serve as a predictive factor for the outcome of GBM patients aged less than 60 years, following alkylating agent chemotherapy [12, 13], or a prognostic factor in non-elderly GBM patients [14]. Compared with other assays, like immunohistochemistry with poor inter-observer reliability and time-consuming procedure, direct testing status of MGMT promoter methylation might be convenient for clinical application. Varying quantitative and qualitative assays, such as MSP, methylation-sensitive high-resolution melting and PSQ, and bisulfite sequencing [15] have been used to examine the methylation status of CpGs island that mainly regulates MGMT protein expression at the epigenetic level, in MGMT promoter. Among these techniques, PSQ is a sequence-by-synthesis method that is the only method respectively analyzing methylation levels of each CpGs and providing quantitative information on the percentage of CpGs methylation [16].

Thus, to our knowledge, this is the first meta-analysis that has evaluated the role of MGMT promoter methylation in predicting the prognosis of GBM patients. In this meta-analysis, because of the prognostic value of methylation status of MGMT promoter by PSQ for survival of GBM patients unclear and no in consensus, we summarized relevant data to quantify the prognostic value of methylation status of MGMT promoter by PSQ, using standard meta-analysis techniques, regardless of impact factors, such as age of patients, therapy modality, etc.

The article "The prognostic value of MGMT promoter status by pyrosequencing assay for glioblastoma patients’ survival: a meta-analysis" was published in 2016. Journal: World J Surg Oncol.

## Methods

We carried out review and meta-analysis following the Cochrane Handbook of systematic reviews and reported results on the basis of Preferred Reporting Item for Systematic Reviews and Meta-Analysis (PRISMA) statement.

### Literature screening

For obtaining a maximum of interested studies, we retrieved literatures in MEDLINE, EMBASE, and Cochrane library (as of Jan. 2016) using the following searching strategy: “(glioblastoma OR glioma) AND (MGMT OR O6-methylguanine-DNA methyltransferase) AND methylation”. It was performed with English restriction and limited to human studies.

### Study selection

The publications were firstly screened by title and abstract by two reviewers, and substantially full-text of potentially eligible studies was reviewed for potential studies under definitive inclusion criteria. Inclusion criteria: (1) studies published the correlation between methylation status of MGMT promoter by PSQ and patients’ outcome; and (2) available data of HR and 95 % CI or *p* value for OS as primary outcome or PFS among GBM patients were extracted, irrespectively of the threshold of methylation status of MGMT promoter the amount of CpGs islands measured by PSQ, disease stage, treatment strategy (whether or not treated with alkylating agent chemotherapy), sample source, etc. Any disagreement or discrepancies were resolved by discussion between less than three reviews.

### Data extraction

From eligible publications, general profiles, like the name of the first author, publication year, country, age of patients, the number of patients, cut-off value of methylation status of MGMT promoter by PSQ, sample source, and treatment experience, as well as disease status, were extracted through two independent reviewers. HRs that were correlated with methylation status of MGMT promoter by PSQ and survival of GBM patients (OS or PFS as outcome) were extracted in multivariate analysis and pooled.

### Assessment of methodological quality

In the context of the Newcastle-Ottawa scale (NOS), which consists of eight items that are categorized into three groups (selection, comparability, and outcome/exposure), two reviewers were involved to assess the methodological quality of eligible studies. Studies with scores of 1–3, 4–6, and 7–9 were considered as low, intermediate, and high quality, respectively.

The article "The prognostic value of MGMT promoter status by pyrosequencing assay for glioblastoma patients’ survival: a meta-analysis" was published in 2016. Journal: World J Surg Oncol.

### Data analysis

For correlation between the status of MGMT promoter methylation by PSQ and patients’ survival, HRs were computed and pooled from each included studies in two cohorts. The fixed-effects or random-effects models were chosen depending on heterogeneity between included studies (assessed by the *I* ^*2*^ statistic test). The *I* ^*2*^ values of 0 to 40 %, 30 to 60 %, 50 to 90 %, and 75 to 90 % indicate no important, moderate, substantial, and considerable heterogeneity, respectively [17]. For significant heterogeneity of studies, we attempted to identify the sources of variation between studies by analyzing the subgroup results and excluding them. Finally, random-effects model was used to pool the results. Because of the amount limitation of eligible studies, sensitivity and publication bias was not undertaken. In this meta-analysis, *p* value was transformed into 95 % CI through formulas [18].

In the two-tailed test, the results were considered to be statistically significant with a *p* value of <0.05. The meta-analysis was performed with Stata 11.0 (Stata Corporation, College Station, Austin, TX).

All analyses were based on the previous published studies; thus, no ethical approval and patient consent were required.

## Results

### Study selection and ascertainment

Using our searching strategy, 2819 publications were found from three database, PubMed-MEDLINE, EMBASE, and Cochrane library. Following reviewing titles and abstracts, 2601 publications were excluded and 218 candidates were included for further assessment. Among these 218 potential publication candidates, ten eligible publications which reported results of 11 studies, all being observational study, were chosen and could successfully extract data for meta-analysis, after excluding review, letter care report, no interesting reports in publication. Flowchart of identification for eligible studies was shown in Fig. 1.

**Fig. 1:** The flowchart of publication search and selection of eligible studies

### Basic characteristic and quality assessment of eligible studies

The main characteristic of the eligible studies was shown in Table 1. All the included 11 prospective cohort studies investigated the association between methylation status of MGMT promoter by PSQ and GBM patients’ survival and reported HR for OS. Of these, four studies presented HR for PFS [19–22]. The age of GBM patients enrolled in the 11 studies ranged widely. In five studies [19, 22–25], 10 % was referred as the cut-off value of the presence of MGMT promoter methylation, 9 % in four studies [26–28], and 8 % in two studies [20, 21]. The amount of CpGs tested by PSQ did not reach an agreement in eligible studies, but at least five CpGs were measured. Of the 11 included studies, not all GBM patients were treated with alkylating agent in three studies [23–25, 28].

The article "The prognostic value of MGMT promoter status by pyrosequencing assay for glioblastoma patients’ survival: a meta-analysis" was published in 2016. Journal: World J Surg Oncol.

**Table 1:** The profiles of eligible studies

Publication year	Study	Country	Age of patient Mean (range or standard derivation)	Cut-off value by PSQ	CpGs	Sample source	No. patients^a^	Disease status	Treatment experience	Score in NOS
2015	Dae Cheol Kim	Korea	51.4 (26.4–87.2)	9 %	5 CpGs	FFPE	104	Newly diagnosed GMB	No all patients treated with TMZ	5
2015	Robert W. Rapkins^b^	Australia	58.3 (25.0–85.0)	9 %	5 CpGs	FFPE	303	Newly diagnosed GMB	Surgery + radiotherapy + TMZ+ adjuvant TMZ	6
2015	Robert W. Rapkins^b^	Australia	57.8 (22.3–84.3)	9 %	5 CpGs	FFPE	303	Newly diagnosed GMB	Surgery + radiotherapy + TMZ+ adjuvant TMZ	5
2014	Veronique Quillien	France	58 (21.0–73.0)	9 %	16 CpGs	FFPE	89	Newly diagnosed GMB	Stupp protocol	5
2014	Vincent Peter Collins	UK	53 (41–60)	10 %	16 CpGs	FFPE	275	Recurrent high-grade GMB	PCV OR two TMZ schedules	5
2014	Dong Shen	China	56 (35–71)	10 %	12 CpGs	FFPE	128	Recurrent high-grade GMB	Surgery + radiotherapy + TMZ+ adjuvant TMZ	5
2012	Guido Reifenberge	Germany	74.1 (70.0–86.6)	8 %	5 CpGs	Frozen sample	85	Newly diagnosed GMB	Treated with alkylating agents	5
2012	Veronique Quillien	France	57.5 (21.0–73.0)	8 %	5 CpGs	FFPE and frozen sample	99	Newly diagnosed GMB	Standard care treatment	5
2011	Miyuki Uno	Brazil	50.2 (14.6)	10 %	5 CpGs	Frozen sample	29	Newly diagnosed GMB	Adjuvant radiotherapy and/or chemotherapy (carmustine)	5
2011	Shani Mulholland	Sweden	NA	10 %	16 CpGs	Frozen sample	362	GMB	Surgery + adjuvant treatment (no TMZ)	5
2009	J Dunn	UK	55 (18–68)	10 %	12 CpGs	FFPE or frozen sample	108	Newly diagnosed GMB	Surgery + radiotherapy + TMZ+ adjuvant TMZ	5

*Abbreviations*: *FFPE* formalin-fixed paraffin-embedded, *PCV* chemotherapy procotol: procarbazine, CCNU, and vincristine

^a^The number of patients whose methylation status of MGMT promoter was measured successfully by PSQ

^b^This publication included two independently studies, Australian cohort (AGOG) and American cohort (UCLA)

In the context of Newcastle-Ottawa quality assessment scale (NOS), the mythological quality of eligible publications was evaluated by two reviewers. The methodological quality of the included 11 studies was evaluated to be intermediate with the score range of 5–6 points, and no study obtained full marks. In category selection, four items, such as representativeness of the exposed cohort, selection of the non-exposed cohort, ascertainment of exposure, and demonstration that outcome of interest, were fully depicted in the 11 studies. In comparability, no control of confounding factors was reported in the 11 eligible studies with all studies scoring 0 point. Only one study depicted that researchers were independently blinded to assess MGMT status by PQS and patients outcomes, and finally, follow-up duration and losses of subjects were not described in all studies (shown in Table 1).

The article "The prognostic value of MGMT promoter status by pyrosequencing assay for glioblastoma patients’ survival: a meta-analysis" was published in 2016. Journal: World J Surg Oncol.

### Overall survival

HR and 95 % CI could be extracted or calculated from *p* value. In this meta-analysis, HRs for OS were analyzed and summarized from three subgroups in which 8, 9, or 10 % as cut-off value was carried out to consider the presence of MGMT promoter methylation in the 11 studies.

In general, MGMT promoter methylation was associated with an HRs for improved OS of 0.50 (95 % CI 0.35–0.66) with statistical heterogeneity (*I* = 84.5 %, *p* = 0.000, random-effects model). The results of subgroup analysis showed that subgroup classification could not reduce heterogeneous level with the value of *I* no less than 85 % (Fig. 2).

**Fig. 2:** Forest plots of the association of methylation status of MGMT promoter by PSQ with OS among GBM patients

After rejecting the data from four studies in which no all patients undergoing alkylating agent chemotherapy, general HRs was 0.42 (95 % CI 0.31–0.53) with statistical heterogeneity (*I* = 67.8 %, *p* = 0.005). In addition, in subgroup 9 %, no obvious heterogeneity was evidenced (*p* < 0.05), and heterogeneity was still in existence in subgroup 10 and 8 % (Fig. 3).

**Fig. 3:** Forest plots of the association of methylation status of MGMT promoter by PSQ with OS among GBM patients after deleting data from four studies in which no all patients treated with alkylating agent

### Progression-free survival

For HRs of PFS, data from four studies were used in meta-analysis, and no subgroups were classified because of limited amounts of eligible studies. Following pooling results in random-effects model, the GBM patients with methylated MGMT promoter had a significantly longer PFS (HR = 0.56, 95 % CI = 0.32–0.80) compared with un-methylated MGMT promoter with statistic heterogeneity (*I* = 80.6 %, *p* = 0.001) (shown in Fig. 4).

**Fig. 4:** HRs for PFS with methylated-positive versus un-methylated cohorts

## Discussion

According to profiling studies of GBM by The Cancer Genome Atlas (TCGA) project, varying subtypes with unique biological behaviors, were identified, such as proneural, neural, classical, and mesenchymal [29] or proneural, proliferative, and mesenchymal [30]. In the context of subtypes by TCGA, Brennan CW et al. found that MGMT promoter status distinguished responders from non-responders to TMZ among samples classified as classical but not among samples classified as proneural, mesenchymal, and neural, evidencing that MGMT promoter methylation might only have such predictive validity in classical subtype GBM [31]. The high rate of MGMT promoter hypermethylation was found long-term GBM survivors that would be of the proneural subtype [32]. In addition, despite methylated-positive MGMT promoter has been recognized with predictive value for ≤60-year-old GBM patients treated with TMZ [12, 13] and prognostic value in non-elderly GBM patients [14], the results are controversial between different studies. The reasons for inconsistency in the results might be that statistical limitation (e.g., small sample size), difference ethnicity of involved subjects, or methodological diversity (e.g., the amount of CpGs detected by PSQ or cut-off value for methylated positivity or tumor sample source). Therefore, the meta-analysis of combining the results from different studies can present direct and definite evidences. Meanwhile, expanding sample-size in the context of homogeneity among including studies in meta-analysis might increase statistical power.

The article "The prognostic value of MGMT promoter status by pyrosequencing assay for glioblastoma patients’ survival: a meta-analysis" was published in 2016. Journal: World J Surg Oncol.

In current meta-analysis, subgroup analysis based on varied cut-off value of MGMT promoter methylation was preformed to address abovementioned issues, and further provide up-to-date clinical evidence for applying MGMT promoter methylation by PSQ as a prognostic biomarker for GBM patients. The result of this meta-analysis showed that, compared with patients with non-methylated MGMT promoter, methylated-positive patients had longer OS and PFS. However, statistical heterogeneity among studies that reported HRs of OS or PFS was observed. Because of adopted varied cut-off value ranged from 8 to 10 % for methylation positivity of MGMT promoter in included studies, three subgroups with cut-off value 10, 9, and 8 % were divided, and then subgroup analysis was undertook according to cut-off value in order to identify the association between the cut-off value and heterogeneity, but the significant heterogeneity was still found. In addition, following simply rejecting data from four studies in which no all GBM patients treated with alkylating agent or from two studies enrolling recurrent GBMs patients, obvious heterogeneity was still in existence. Therefore, the cut-off value of MGMT promoter positivity with PSQ and therapy modality might not be the main reason for high level of heterogeneity in this meta-analysis. Other factors, such as sample size, age, and follow-up duration were investigated, but no heterogeneous sources were identified.

Methylation of CpGs sites in MGMT promoter, one of the major post-transcriptional mechanisms reducing MGMT protein expression, has been found in 40 % of cancer such as glioma and colorectal cancer and in 25 % of non-small cell lung carcinoma, lymphoma, and head and neck carcinoma [33, 34]. Furthermore, the extent of methylation has an impact on the expression levels of MGMT protein [35]. Thus, it is mechanistically reasonable that the methylation status of MGMT promoter might be regarded as a prognostic biomarker for GBM patients treated with alkylating agent. In comparison with other assay, PSQ yields quantitative results, and high intra- and inter-laboratory reproducibility for a commercially available MGMT PSQ kit is documented in a ring trial [36]. However, standard operation procedure of PSQ should be established, and accuracy should be determined soon.

The article "The prognostic value of MGMT promoter status by pyrosequencing assay for glioblastoma patients’ survival: a meta-analysis" was published in 2016. Journal: World J Surg Oncol.

There were some limitations in this meta-analysis. Firstly, the number of eligible studies included was limited, and outcome measures recorded differently in the studies. Especially, only four studies were involved for PFS, so the results should be interpreted with cautions. Secondly, statistical heterogeneity among these studies that reported HR for OS and PFS were observed, and the source of heterogeneity were not able to be determined simply by subgroup analysis on the basis of the cut-off value of MGMT promoter methylation by PSQ or rejecting data from four studies in which no all patients underwent alkylating agent chemotherapy. Thirdly, due to limited number of studies included in this meta-analysis, sensitivity analysis and publication bias were not been evaluated. Fourthly, the cohort studies included in this meta-analysis had an intermediate methodological quality with no more than 6 points in NOS, so there were some methodological issues. Lastly, although Karnofsky performance score, age, sex, etc. were analyzed as potential prognostic factors in multivariate analysis in the 11 eligible studies, no studies in this meta-analysis explained the control of confounding factors.

## Conclusions

In spite of above limitations, our meta-analysis indicated that the methylation status of MGMT promoter were related to the improved prognosis by PSQ and should be considered as a strong prognostic biomarker among GBM patients post-TMZ therapy. According to methylation status by PSQ, stratification medication might be applied among GBM patients in coming clinical practice.

## Abbreviations

CI: Confidence interval
GBM: Glioblastoma
HRs: Hazard ratios
MGMT: O^6^-Methylguanine-DNA methyltransferase
NOS: Newcastle-Ottawa scale
OS: Overall survival
PFS: Progression-free survival
PSQ: Pyrosequencing assay
TMZ: Temozolomide
